# Leaf Rolling and Stem Fasciation in Grass Pea (*Lathyrus sativus* L.) Mutant Are Mediated through Glutathione-Dependent Cellular and Metabolic Changes and Associated with a Metabolic Diversion through Cysteine during Phenotypic Reversal

This article has been retracted.

**DOI:** 10.1155/2014/479180

**Published:** 2014-05-28

**Authors:** Dibyendu Talukdar, Tulika Talukdar

**Affiliations:** ^1^Department of Botany, R.P.M College, University of Calcutta, Uttarpara, Hooghly, West Bengal 712 258, India; ^2^Department of Botany, Acharya Prafulla Chandra Roy Government College, University of North Bengal, Darjeeling, West Bengal 734 010, India

## Abstract

A *Lathyrus sativus * L. mutant isolated in ethylmethane sulfonate-treated M_2_ progeny of mother variety BioL-212 and designated as *rlfL-1* was characterized by inwardly rolled-leaf and stem and bud fasciations. The mutant exhibited karyomorphological peculiarities in both mitosis and meiosis with origin of aneuploidy. The mitosis was vigorous with high frequency of divisional cells and their quick turnover presumably steered cell proliferations. Significant transcriptional upregulations of cysteine and glutathione synthesis and concomitant stimulations of glutathione-mediated antioxidant defense helped *rlfL-1* mutant to maintain balanced reactive oxygen species (ROS) metabolisms, as deduced by ROS-imaging study. Glutathione synthesis was shut down in buthionine sulfoximine- (BSO-) treated mother plant and mutant, and leaf-rolling and stems/buds fasciations in the mutant were reversed, accompanied by normalization of mitotic cell division process. Antioxidant defense was downregulated under low glutathione-redox but cysteine-desulfurations and photorespiratory glycolate oxidase transcripts were markedly overexpressed, preventing cysteine overaccumulation but resulted in excess H_2_O_2_ in BSO-treated mutant. This led to oxidative damage in proliferating cells, manifested by severe necrosis in rolled-leaf and fasciated stems. Results indicated vital role of glutathione in maintaining abnormal proliferations in plant organs, and its deficiency triggered phenotypic reversal through metabolic diversions of cysteine and concomitant cellular and metabolic modulations.

## 1. Introduction

Intracellular thiol redox status is a critical parameter in determining plant growth and development in response to continuous production of reactive oxygen species (ROS) [1]. In aerobic cells, ROS homeostasis is delicately balanced [2, 3] and mediates crucial intracellular signaling pathways which are essential for cell survival [3]. However, an excess of ROS formation shifts the redox balance in favor of oxidative state which leads to cell damage and death. The increase of ROS, however, can induce an adaptive response, consisting of a compensatory upregulation of antioxidant systems, aimed to restore the redox homeostasis [3, 4]. Glutathione (reduced form: GSH; oxidized form: GSSG), the tripeptide *γ*-glutamylcysteinylglycine, is the principal antioxidant component and predominant form (>90%) of nonprotein thiol within a cell. In plants, GSH is synthesized enzymatically from its constituent amino acids via two-step ATP-dependent pathway catalyzed by *γ*-glutamylcysteine synthetase (*γ*-ECS), the rate-limiting step, and can be inhibited by treating with BSO (L-buthionine sulfoximine) and GSH synthetase (GSHS) [3]. Owing to the presence of a strong nucleophilic thiol group on its cysteine (Cys) residue, GSH interacts with numerous cellular components as an efficient redox buffer, provides valuable information on cellular redox state, and, most importantly, regulates enzymatic processes both upstream of thiol-cascade and downstream of thiol metabolites in order to maintain plant growth and maximize cellular defenses against stresses [1, 3]. GSH is an important factor controlling cell proliferations during tumour growth in animal cells [5]. Elevated GSH levels were observed in various types of proliferative response and progression of cell cycle [5]. Moreover, the content of GSH in some tumor cells is typically associated with higher levels of GSH-related enzymes, such as *γ*-ECS activities [5]. In plants, GSH is crucial in postembryonic development of the root [6] and the shoot [3], but despite many morphological and biochemical features similar to those found in animal cells, evidence for thiol involvement in plant tumorigenesis is not convincing [7]. GSH plays central role in regeneration of reduced ascorbate from its oxidized form dehydroascorbate (DHA). The resultant glutathione disulfide or GSSG is then recycled to GSH by NADPH-dependent action of glutathione reductase (GR) in ascorbate-GSH cycle [3]. The reduced ascorbate is used as an exclusive cofactor by ascorbate peroxidase during scavenging of H_2_O_2_ [3]. The H_2_O_2_ is one of the prominent diffusible ROS within the cell and is continuously generated in aerobic cells by photorespiration, activity of superoxide dismutase (SOD), and other reasons. Dual roles of H_2_O_2_ as an inducer of oxidative stress and a powerful signaling molecule for antioxidant upregulations have been investigated in crop plants, experiencing biotic and abiotic stresses [8–11]. The conjugation of GSH to heavy metals, herbicides, and xenobiotics is accomplished by multifunctional enzymes glutathione* S*-transferases (GSTs) [12], establishing the now widely accepted role of GSTs as cell housekeepers involved in the detoxification of endogenous as well as exogenous substances. More recently, several GST isoenzymes have been shown to modulate cell signaling pathways that control animal cell proliferation and cell death (apoptosis) [5, 13]. Blockage of the GSH/GST detoxification system enhanced the chemosensitivity of several tumor cell lines. Consequently, excess generation of oxidative intermediates and depletion of GSH have been found to either precede the onset of apoptosis or render the cells more sensitive to death [5, 13]. Glutathione peroxidases (GPXs) are also involved in removal of organic peroxides and H_2_O_2_ using GSH or thioredoxins as electron donors [3]. The GSH/(GSH + GSSG) ratio, considered as GSH redox state, is likely to be far more influential in the antioxidant defense, controlling gene expressions and thionylation process than the absolute size of the glutathione pool [3].

Cysteine (Cys), one of the vital building blocks of GSH, is the first stable and committed molecule in plant metabolism that contains both sulfur and nitrogen, synthesized by the O-acetylserine (thiol)lyase (OAS-TL) either in free active homodimer or in association with serine acetyltransferase (SAT) as an inactive subunit of the cysteine synthase complex [1, 14]. OAS-TL is the most enigmatic enzymatic systems in sulfur metabolisms and its isoforms along with SAT in different cellular compartments are under strict regulations in plants responding to environmental stresses [1, 14, 15]. While depleting Cys level escalates the stress sensitivity [1, 15], free Cys, but not GSH, above a certain concentration threshold reportedly has the ability to exacerbate the prooxidant properties due to high reactivity of its thiol moiety [16, 17]. The opposite mechanisms of Cys biosynthesis and its cellular degradation have immense significance in maintaining Cys homeostasis and this is under tight regulations under stressful environments [16–18]. Studies indicate that Cys degradation is mainly mediated through the desulfuration of L-Cys and D-Cys by L-cysteine desulfhydrase (LCD) and D-cysteine desulfhydrase (DCD), respectively, rather than promoting Cys biosynthesis in high plants [18]. The resultant hydrogen sulfide participates in different physiological activities to promote plant growth processes but can also induce oxidative stress to promote cell death [18–20].

Development of plant organ is highly dynamic and involves the controlled initiation of new primordia from groups of stem cells called meristems. Leaves and the axillary meristems that generate branches and flowers are initiated in regular patterns under tight cellular regulations from the shoot apical meristem (SAM), balancing cell proliferation with the incorporation of cells into new primordia [21]. This balance is essential to maintain SAM integrity and the stereotypical pattern of organ initiation throughout development. Leaf rolling and stem proliferation are two important phenomena in plant developmental process [22–24]; while leaf rolling is supposed to be an adaptation to drought tolerance mechanisms, proliferative growth in stems, buds, and in other plant organs often leads to fasciation through disturbances in SAM. Although moderate leaf rolling and fasciation in plant parts have long been utilized for crop yield enhancement [22], they are still regarded as an enigmatic process as nothing is known regarding intrinsic cellular and biochemical processes involved in cell proliferations during rolling and fasciation. Most of the studies in shoot meristem proliferation have come from mutations in* Arabidopsis* such as* clavata*,* mgoun1 *and* mgoun2*,* fasciata1 *and* fasciata2*, and* fully fasciated *[23] and in maize [24], revealing involvement of genetic events in the process. To date, 12 rice mutants with rolled leaves have been isolated [22]. However, despite immense importance of leaf rolling and stem fasciation in cell physiological and agronomic point of view and roles of GSH-redox status in regulation of plant growth events, scanty work has been done in this direction [25]. Also, no reports are available regarding cytogenetic behavior of proliferative vegetative and reproductive cells in plants. Grass pea is a very hardy cool-season legume crop, used both for food and feed worldwide. The novelty of this crop in cell biology research has been manifested through development of robust cytogenetic and mutation stocks to decipher the cellular and metabolic events leading to plant growth, development, and stress tolerance [26–28]. Here, we isolated one unique grass pea mutant, exhibiting characteristic leaf-rolling and stem as well as axillary bud fasciation, in M_2_ progeny of ethylmethane sulfonate- (EMS-) mutagenized population. The mutant was advanced to next generation through self-pollination to perform a detail study. The main goal of the present investigation was to trace the intrinsic cellular and GSH-mediated mechanisms behind the phenotypic abnormalities in the mutant plants with the objectives to (1) measure the Cys and GSH pool, (2) investigate the activities and mRNA gene expressions of Cys and GSH biosynthesis and GSH-dependent antioxidant systems, (3) assess the mitotic fidelity and chromosomal anomalies, and (4) detect the ROS accumulation and oxidative damage in untreated and BSO-treated tissues of mother variety and mutant line.

## 2. Materials and Methods

### 2.1. Induction and Detection of Mutants

Fresh seeds of grass pea (*Lathyrus sativus *L. cv. BioL-212) were collected from Pulses and Oilseed Research Station, Berhampore, West Bengal, India, and grown for two seasons (2010 and 2011) in a private farm at Kalyani (22°59′N/88°29′E), West Bengal, India. After ascertaining uniformity of seed age and homozygosity, fresh seeds presoaked in water for 5 h were treated with freshly prepared 0.15%, 0.25%, and 0.5% aqueous solution of ethylmethane sulfonate (EMS) for 6 h with intermittent shaking at 25 ± 2°C keeping a control (distilled water). After the stipulated period, seeds were thoroughly washed with running tap water and sown in the field treatment wise (200 seeds treatment^−1^) along with untreated seeds as control in triplicate during November 2012 (temperature 20°C/18°C, day/night, relative humidity 72 ± 4%, photoperiod 10 h, irradiance 180–200 *μ*mol m^−2^ s^−1^). Selfed seeds of individual M_1_ plants were harvested separately and were grown in the next season in a randomized block design keeping a distance of 30 cm between rows and 20 cm between plants to raise M_2_ progeny. Standard agronomic practices were followed to grow healthy plant progeny. Phenotypes of about 2000 M_2_ individuals were screened during winter of 2012 and 2013. One plant with characteristic in-rolled leaflets and proliferation in stem and axillary buds has been isolated in M_2_ progeny of EMS- (0.25%, 6 h) treated population. Seeds (42 seeds) of this variant plant were carefully harvested and sown in the next season to raise M_3_ progeny. The mutant phenotype was true breeding, and based on morphological peculiarities, the mutant was designated as* rlfL-1* (*Rolled leaflet and fasciated Lathyrus mutant-1*). Further biochemical and molecular characterizations of the mutant were performed on these progeny plants.

### 2.2. Culture Conditions and BSO Treatment Protocol

Grass pea seeds obtained from M_3_ plants of* rlfL-1* mutant and its mother variety BioL-212 were surface-sterilized with 70% ethanol for 2 min, rinsed twice in deionized water, and then placed on water-moistened filter papers at dark to germinate at 25°C. Germinated seedlings were immediately placed in polythene pots (10 plants pots^−1^) containing 300 mL of Hoagland's number 2 nutrient media and were permitted to grow for 10 d. The media were either unsupplemented (control plants) or supplemented (three treatment sets) with 1 mM BSO (L-buthionine sulfoximine, Sigma-Aldrich, Bangalore, India) and the seedlings were allowed to grow for another 5 d. Mother variety and* rlfL-1 *plants submitted to untreated (0 mM BSO) condition were used as mother control (MC) and mutant control (MuC), respectively, while those treated with BSO were designated as treated mother (TM) and treated mutant (MuT), respectively. Plants were harvested at 15 d growth period. The experiment was carried out in a completely randomized block design with three replicates in an environmentally controlled growing chamber under a 14-hour photoperiod, temperature of 28/18 ± 2°C, relative humidity of 70 ± 2%, and a photon flux density of 100 *μ*mol m^−2^ s^−1^. Shoots and roots were rinsed thoroughly with sterile distilled water and oven-dried at 65°C for 72 h to weigh dry mass.

### 2.3. Estimation of Glutathione, Cys, and Assay of Thiol Metabolizing Enzymes

Reduced and oxidized forms of glutathione were measured following the methods of Griffith [29]. For enzyme assay, plant tissue (leaves and stems) was homogenized in buffers specific for each enzyme under chilled conditions. The homogenate was squeezed through four layers of cheese cloth and centrifuged at 12,000 g for 15 min at 4°C. The protein content of the supernatant was measured using BSA as standard [30]. Assay of serine acetyltransferase (SAT; EC 2.3.1.30) activity was performed following Blaszczyk et al. [31]. An enzyme unit was considered as the amount of enzyme catalyzing the acetylation of 1 pmol of L-serine per minute. The OAS-TL (EC 2.5.1.47) activity was assayed by measuring the production of L-Cys. Assay was started by the addition of 5 *μ*L crude extract (1 *μ*g *μ*L^−1^ total protein in 50 mM phosphate buffer, pH 8.0). Reactions were conducted in 50 mM phosphate buffer (pH 8.0) in the presence of 5 mM dithiotreitol (DTT), 12.5 mM O-acetyl L-serine (OAS), and 4 mM sodium sulfide (Na_2_S) in a total volume of 100 *μ*L assay mixture and allowed to proceed for 30 min at 30°C. The reaction was terminated by the addition of 0.1 mL of 7.5% trichloroacetic acid [32]. Cys content was measured spectrophotometrically (Perkin-Elmer, Lambda 35, Mumbai, India) at 560 nm following Gaitonde [33]. A blank control with all compounds except OAS was maintained, and the linearity of the assay was checked with 2.5 and 10 *μ*L of added crude leaf extract. Assay of *γ*-ECS (EC 6.3.2.2) and LCD (EC 4.4.1.1) was done by following Seelig and Meister [34] and Bloem et al. [35], respectively. LCD (EC 4.4.1.1) activity was measured by the release of sulfide from Cys in a total volume of 1 mL consisting of 2.5 mM dithiothreitol, 0.8 mM L-Cys, 100 mM TRIS/HCl, pH 9.0, and enzyme extract [35]. The reaction was initiated by the addition of L-Cys. After incubation for 15 min at 37°C the reaction was terminated by adding 100 *μ*L of 30 mM FeCl_3_ dissolved in 1.2 N HCl and 100 *μ*L of 20 mM N,N-dimethyl-p-phenylenediamine dihydrochloride dissolved in 7.2 N HCl [35]. The formation of methylene blue was determined at 670 nm. Solutions with different concentrations of Na_2_S were prepared and treated in the same way as the assay samples and were used for the quantification of enzymatically formed H_2_S. DCD (EC 4.4.1.15) activity was determined in the same way, but D-Cys was used instead of L-Cys [35]. Four samples per treatment were collected with four replications in the assays.

### 2.4. Assay of Antioxidant Enzymes

Tissue of 250 mg was homogenized in 1 mL of 50 mM K-phosphate buffer (pH 7.8) containing 1 mM EDTA, 1 mM DTT, and 2% (w/v) polyvinyl pyrrolidone using a chilled mortar and pestle kept in an ice bath. The homogenate was centrifuged at 15,000 g at 4°C for 20 min. Clear supernatant was used for enzyme assays. For measuring APX activity, the tissue was separately ground in homogenizing medium containing 2.0 mM AsA in addition to the other ingredients. All assays were done at 25°C. Soluble protein content was determined using BSA as a standard [30]. SOD (EC 1.15.1.1) activity was determined by the nitro-blue tetrazolium (NBT) assay as described by Beyer Jr. and Fridovich [36] and detailed earlier [37]. For ascorbate peroxidase (APX, EC 1.11.1.11) activity, three milliliter of the reaction mixture contained 50 mM potassium phosphate buffer (pH 7.0), 0.1 mM EDTA, 0.5 mM ascorbate, 0.1 mM H_2_O_2_, and 0.1 mL enzyme extract. The H_2_O_2_-dependent oxidation of ascorbate was followed by a decrease in the absorbance at 290 nm (extinction coefficient 2.8 mM^−1 ^cm^−1^). APX activity was expressed as *μ*mol ascorbate oxidized min^−1 ^mg^−1^ protein [38]. GR (EC 1.6.4.2) activity was determined by monitoring the GSH-dependant oxidation of NADPH, as described by Carlberg and Mannervik [39]. In a cuvette, 0.75 mL 0.2 M potassium phosphate buffer (pH 7.0) containing 2 mM EDTA, 75 *μ*L NADPH (2 mM), and 75 *μ*L oxidized glutathione (20 mM) were mixed. Reaction was initiated by adding 0.1 mL enzyme extract to the cuvette and the decrease in absorbance at 340 nm was monitored for 2 min. GR-specific activity was expressed as nmol NADPH oxidized min^−1 ^mg^−1^ protein. GST (EC 2.5.1.18) activity was assayed in a reaction mixture containing 50 mM phosphate buffer, pH 7.5, 1 mM 1-chloro-2,4-dinitrobenzene (CDNB), and the elute equivalent to 100 *μ*g of protein. The reaction was initiated by the addition of 1 mM GSH (Sigma-Aldrich), and formation of S-(2,4-dinitrophenyl) glutathione was monitored as an increase in absorbance at 334 nm to calculate the GST-specific activity [40]. Total GPX (EC 1.15.1.1) activity was determined from 1 g plant tissues extracted in 3 mL of 0.1 M Tris-HCl, pH 7.5, containing 2 mM DTT and 1 mM EDTA. The enzyme activity was ascertained by using cumene hydroperoxide (both selenium and nonselenium enzyme types) as a substrate and GR coupled assay to monitor the oxidation of GSH [41]. GPX activity was expressed as change in absorbance at 340 nm. Glycolate oxidase (GO; EC 1.1.3.15) activity was assayed by the formation of a glyoxylate-phenylhydrazone complex at 324 nm [42]. The GO assay mixture contained 100 mM of phosphate buffer (pH 8.3), 40 mM glycolic acid, 100 mM L-Cys, and 100 mM phenylhydrazine. The reaction was started with the addition of the 1 mM FMN, and the absorbance was monitored over 300 s. GO activity was calculated using the molar extinction coefficient of the glyoxylate-phenylhydrazone complex (17 mM^−1 ^cm^−1^) and was expressed as *μ*mol glyoxylate min^−1 ^mg^−1^ protein.

### 2.5. Measurement of Endogenous H_2_S

Endogenous H_2_S was determined by the formation of methylene blue from dimethyl-p-phenylenediamine in H_2_SO_4_ [19, 43], with some modifications. About 0.5 g of tissues was ground and extracted in 5 mL of phosphate buffer solution (pH 6.8, 50 mM) containing 0.1 M EDTA and 0.2 M ascorbate. The homogenate was mixed with 0.5 mL of 1 M HCl in a test tube to release H_2_S, and H_2_S was absorbed in a 1% (w/v) zinc acetate (0.5 mL) trap, located in the bottom of the test tube. After 30 min of reaction, 0.3 mL of 5 mM dimethyl-p-phenylenediamine dissolved in 3.5 mM H_2_SO_4_ was added to the trap. Then 0.3 mL of 50 mM ferric ammonium sulfate in 100 mM H_2_SO_4_ was injected into the trap. Amount of H_2_S in zinc acetate traps was determined spectrophometrically at 667 nm after leaving the mixture for 15 min at room temperature. Blanks were prepared by the same procedures without the zinc acetate solution.

### 2.6. Determination of H_2_O_2_ Content, Lipid Peroxidation Level, and Electrolyte Leakage %

Level of H_2_O_2_ was estimated following the methods of Wang et al. [44]. Fresh tissue of 0.1 g was powdered with liquid nitrogen and blended with 3 mL acetone for 30 min at 4°C. Then the sample was filtered through eight layers of gauze cloth. After addition of 0.15 g active carbon, the sample was centrifuged twice at 3,000 g for 20 min at 4°C; then 0.2 mL 20% TiCl_4_ in HCl and 0.2 mL ammonia were added to 1 mL of the supernatant. After reaction, the compound was centrifuged at 3,000 g for 10 min; the supernatant was discarded and the pellet was dissolved in 3 mL of 1 M H_2_SO_4_ and absorbance was measured at 410 nm. H_2_O_2_ content was measured from the absorbance at 410 nm using a standard curve [44]. Lipid peroxidation was determined by measuring the malondialdehyde (MDA) equivalents while EL% was assayed following the methods detailed earlier [45].

### 2.7. Relative Gene Expression Analysis through Quantitative RT-PCR

Candidate mRNA gene expression levels of SAT, OAS-TL, *γ*-ECS, LCD, DCD, SOD, APX, GR, GSTs, GPX, and GO of control (MC and MuC) and BSO-treated plants (TM and MuT) were analyzed by quantitative reverse transcription polymerase chain reaction (qRT-PCR) technique. Total RNA was isolated using the RNA isolation kit (Chromous Biotech, Bangalore, India) and treated with DNaseI (Chromous Biotech, Bangalore, India) at 37°C for 30 min. The quality of total RNA samples was determined spectrophotometrically (Perkin-Elmer, Lambda 35, Mumbai, India) from A260/280 ratio and by 1% agarose gel electrophoresis. First strand cDNA was synthesized from DNA-free intact RNA with oligo-dT primers and with MmuLV reverse transcriptase enzyme kit (Chromous Biotech, Bangalore, India) following manufacturer's instructions. Quantitative RT-PCR of first-strand cDNA was run on ABI Step-One (Applied Biosystems, Foster City, CA, USA) Real-Time PCR machine. Amplification was done in a total reaction volume of 50 *μ*L, containing template (first-strand cDNA) 2.0 *μ*L, forward and reverse primer 2.0 *μ*L each with 50 nM *μ*L^−1^ concentration, 2× PCR SYBR green ready mixture (Fast Q-PCR Master Mix Chromous Biotech, India, cat number QCR 05/QCR 06) 25.0 *μ*L, and DEPC water 19.0 *μ*L. Primers for selected genes were constructed by Primer Express V. 3.0 software (Applied Biosystems, Foster City, CA, USA) with the search of available sequence databases (http://www.ncbi.nlm.nih.gov) and reports on* Phaseolus vulgaris* [37],* Lens culinaris* [15, 46], and* Arabidopsis thaliana* [18, 47]. The sequences (5′→ 3′) of forward (F) and reverse (R) primer in each of the candidate genes are presented in Table 1. The qRT-PCR cycling stages consisted of initial denaturation at 94°C (3 min), followed by 35 cycles of 94°C (5 s), 62°C (10 s), 72°C (10 s), and a final extension stage at 72°C (2 min). A melting curve analysis was performed after every PCR reaction to confirm the accuracy of each amplified product. Samples for qRT-PCR were run in four biological replicates with each biological replicate containing the average of three technical replicates. DEPC water for the replacement of template was used as negative control. RT-PCR reaction mixtures were loaded onto 2% agarose gels in TAE buffer. A 100-bp DNA ladder was run on every gel. The mRNA levels were normalized against* L. culinaris EF1-*α** as the housekeeping gene, and the relative (to control) expression of target genes was calculated as 2^−ΔΔCt^ (http://www.Appliedbiosystems.com/support/apptech/#rtpcr) following Livak and Schmittgen [48].

### 2.8. Cytogenetic Assay

For mitotic study, leaf tips from growing leaves (rolled as well as normal) were pretreated with 2 mM 8-hydroxyquinoline for 2.40 h at room temperature followed by fixation in 45% acetic acid for 15 minutes at 4°C. These were then hydrolyzed in a mixture of 1 N HCL and 45% acetic acid (2 : 1) at 60°C for 10 s. The leaf tips were stained and squashed in 1% aceto-orcein [49]. Mitotic index (MI) was determined by counting the number of mitotic cells among the total number of scored cells and expressed in percentage. Mitotic phase distribution was studied by scoring frequencies of prophase, metaphase, anaphase, and telophase from the same slides where MI was calculated. The phase indices-prophase index (PI), metaphase index (MtI), anaphase index (AI), and telophase index (TI) were determined by calculating the number of cells in the respective phase among the number of total dividing cells and expressed as percentage [49]. In order to ascertain the duration of divisional stages, growing leaf tips (from rolled leaves and MC separately) were fixed sequentially one after another with an interval of 15 min and then were stained and squashed. The fixation time was recorded in each case. Duration of total divisional phases (prophase to telophase) was calculated by scoring particular time of fixation from prophase to telophase. Similarly, duration for particular stage was determined by scoring the fixation times when the respective stages peaked in frequency. Six replicates were maintained for each set. The duration of each mitotic stage can now be calculated using the following equation [50]:

(1) Duration  of  mitotic  stage =Number  of  cells  in  a  particular  stageTotal  number  of  cells×105  minutes

considering that the duration of mitosis from start to finish (including all four stages) is 105 minutes (8.30–10.15 a.m.) in grass pea (Talukdar, unpublished). For each leaf tip sample, 1000 cells were scored, taking note at which stage the cell was in: prophase, metaphase, anaphase, or telophase. Meiotic analysis was carried out following the procedure employed earlier in grass pea [51]. Briefly, suitable sized flower buds collected separately from each genotype were fixed between 9.00 a.m. and 10.00 a.m. in propionic acid alcohol (1 : 2) for 6 h and then were preserved in 70% alcohol for future studies. After washing the fixed buds in distilled water, anthers were smeared in 1% propionocarmine solution to analyze meiosis in the microsporocytes. Photomicrographs were taken from well-scattered plants. Sterility of pollen grains was studied following staining of randomly selected anthers with 1% acetocarmine solution and expressed as percentage [51].

### 2.9. Detection and Imaging of Superoxide and H_2_O_2_ Radicals by Confocal Laser Scanning Microscopy

Detection and imaging of superoxide radicals in leaf and stem sections were carried out using the fluorescence probe dihydroethidium (DHE), following the earlier method [37]. Grass pea leaf and stem segments of approximately 30 mm^2^ were incubated for 1 h at 25°C, in darkness, with 10  *μ*MDHE prepared in 5 mM Tris-HCl buffer at pH 7.4, and samples were washed twice with the same buffer for 12 min each. After washing, leaf sections were embedded in a mixture of 15% acrylamide-bisacrylamide stock solution, and 100 mm thick sections, as indicated by the vibratome scale, were cut under 10 mM phosphate-buffered saline (PBS). Sections were then soaked in glycerol : PBS (containing azide) (1 : 1 v/v) and mounted in the same medium for examination with a (CLSM) system (Carl Zeiss, LSM 780, Bangalore, India) using standard filters and collection modalities for DHE green fluorescence (*λ* excitation 488 nm; *λ* emission 520 nm) and chlorophyll autofluorescence (Chl a and b, *λ* excitation 429 and 450 nm, resp.; *λ* emission 650 and 670 nm, resp.) as blue. H_2_O_2_ was detected by incubation with 25 *μ*M 2′ 7′-dichlorofluorescein diacetate (DCF-DA) (excitation 485 nm, emission 530 nm) [37]. Preinfused leaf and stem sections with 1 mM tetramethylpiperidinooxy (TMP), a scavenger of superoxide radicals, and 1 mM ascorbate, a scavenger of H_2_O_2_, served as negative controls.

### 2.10. Statistical Analysis

The results presented were the mean values ± standard errors obtained from at least four replicates. Statistical significance of mean values between control and treated seedlings was determined by Students* t*-test (two-tailed) using Microsoft Excel tool pack “data analysis” 2007. Multiple comparisons among treatments were performed by ANOVA using software SPSS v. 10.0 (SPS Inc., USA), and means were separated by Duncan's multiple range test. A probability of *P* < 0.05 was considered significant.

## 3. Results and Discussions

### 3.1. Phenotypic and Karyo-Morphological Peculiarities in *rlfL-1* Mutant in Untreated and BSO-Treated Experimental Conditions

The* rlfL-1* mutant exhibited characteristic inwardly rolled (revolute) leaflet pair in compound leaves of grass pea compared to usual linear-lanceolate leaflet pair in MC plants (Figures 1(a), and 1(b)). The rolling of leaflets started from its terminal part since very early seedling stage (Figures 1(c) and 1(d)) and reached in full rolling at vegetative stage much before the onset of flowering (Figure 1(a)). Leaf rolling has been considered as a morphophysiological adaptation of crop plants for drought/heat stress avoidance mechanisms and diseases and or nutritional deficiency [52]. Leaf rolling is orchestrated through abnormal overdivisions of leaflet cells present in the opposite direction of rolling and/or lower divisional rate of cells situated inside the rolling [22, 53–55]. In the present mutant, upper surface of leaflets remained outside during rolling. The present mutant is unique in the sense that the seedlings were quite healthy and possessed higher shoot and root dry weight than MC (Table 2) and no dwarfism as well as stress situation was apparent. The MC of the mutant was largely uniform without any type of leaf rolling. In grass pea, inward leaf coiling has been reported in genotypes possessing aneuploid genomes [26, 51]. Although fasciated stem was reported in grass pea [56, 57], occurrence of both rolling and fasciation in a single plant was isolated for the first time in a diploid genotype of grass pea.

Leaf rolling in* rlfL-1* mutant was intimately associated with appearance of stem and axillary bud fasciation in the present investigation (Figures 2(a) and 2(b)). Fasciation resulting from proliferative growth has been explored as a SAM mutant in plants [21–23]. Among food legumes, stem fasciation was successfully induced by mutagenic techniques in grass pea [56, 57], chickpea [58], soybean [59], lentil, pea, and other plants [60]. In the present case, overgrowth of stem tissue was observed sporadically in association with proliferation in axillary buds. The buds were drooping from axis of the mutant plants (Figure 2(b)). The occurrence of fasciated portions was, however, not uniformly distributed in stems of* rlfL-1* mutant. Importantly, not all leaflets in the mutant were rolled, nor all the axillary buds carried proliferations. Significantly, stem and bud proliferation was noticed in those regions where adjacent leaflet pairs were rolling (Figure 2(b)), and nearly 80% of total leaflets were found rolled. The proliferated buds in* rlfL-1* mutant often developed larger-sized pods with bolder seed and higher 100 seed weight compared to MC. However, the number of seeds per pod reduced (Table 2). Productions of larger-sized seeds are of great commercial importance in legume breeding [61] and suggest partial beneficial effect of present* rlfL-1* mutant in grass pea.

The* rlfL-1* mutant showed cytological peculiarities, as manifested in rolled leaf-tip mitosis and fasciated flower bud meiosis. Compared to 14 chromosomes uniformly distributed in diploid genomes of MC plant and also in normal (MC-like) linear-lanceolate leaflet tip (Figure 3(a)), chromosomes were largely anomalous in rolled leaf-tip of the mutant. The abnormal behavior was characterized by the presence of fragmented chromosomes, unoriented chromosomes, C-mitosis, multipolarity, sticky metaphase, cytomixis, anaphase bridge with or without laggard, broken bridge, diagonal orientations of chromosomes, and aneuploid cells (Figures 3(b)–3(l)). The aneuploid cells were largely trisomics (2*n* = 2*x* + 1 = 15) or double trisomics (2*n* = 2*x* + 1 + 1 = 16) and often unoriented during mitotic metaphase (Figure 3(g)). In meiosis of fasciated bud, nearly 42% of total pollen mother cells (PMCs) exhibited usual pairing of seven bivalents (7 II) with 2*n* = 2*x* = 14 chromosomes (Figure 4(a)). The rest of the cells were aberrant due to presence of multivalent, univalents, unequal separation of anaphase chromosomes, bridges and lagging chromosomes, micronucleus formations, and aneuploids (Figures 4(b)–4(p)). Multinucleolate conditions accompanied with long retention of nucleoli even at anaphase I were also encountered sporadically (Figures 4(c) and 4(d)). The nucleolus is the major centre of controlling protein synthesis, and thus origin of more than one nucleolus and its retention by dividing cells indicates enhanced protein synthesizing capacity required in the fasciated buds. The results agreed well with occurrence of more than one nucleolus per cell in tumorous HNO (habituated nonorganogenic) cell lines of sugar beet, and the polynucleolation has been regarded as a representative feature of very high rate of cellular metabolism, often observed in cancerous cells [7]. The extra chromosomes in trisomics were either in univalent or in trivalents (Figures 4(g), 4(i), 4(j), and 4(l)). Occurrence of “Y”-shaped, frying pan shaped, or rod-shaped trivalents at meiotic metaphase indicated origin of primary trisomics while pentavalent formation at meiosis I suggested existence of trisomic genomes with interchanged chromosomes (Figures 4(f) and 4(l)). Occurrence of diagonal orientation, chromosome stickiness, multipolarity, and unorientation of metaphase chromosomes suggested spindle disturbances in dividing cells both in vegetative and reproductive tissues undergoing abnormal proliferations in* rlfL-1* mutant. Variations in chromosome number accompanied with diverse types of karyological aberrations like aneuploidy, asynapsis, desynapsis, translocation, fragmented chromosomes, univalents, and anaphase bridges, were observed in* Haplopappus gracilis*, crown-gall callus of* Nicotiana tabacum*, hormone-induced tissue of* Pisum sativum*,* Lotus corniculatus*,* Avena sativa*, rice, wheat, and many other plant species [62]. Obviously, anomalous chromosomal associations in meiosis of PMCs resulted in reduction of pollen fertility (43.11%) in proliferated buds but it was still enough to maintain self-fertility of the mutant. In animal cells, aberrant cells are often found in tumor cells and occurrence of fragmented and lagging chromosomes as also observed in the present investigation indicates the risk of aneuploidy and further aberrations [63]. Aneuploidy causes a proliferative disadvantage in all normal cells studied so far; yet this condition is associated with unabated proliferative potential [63]. Occurrence of substantial number of trisomic and double trisomic cells in the present* rlfL-1* mutant suggested origin of extra chromosomes in the diploid complement, bringing about further disturbances in mitosis and meiosis. Furthermore, due to wasteful transcription, translation, and degradation of proteins encoded by extra chromosomes in trisomic genomes and dosage-effects, aneuploidy dramatically increases cell's energy needs and altered metabolisms often generates excess ROS [64]. Although, these factors are generally believed to lower the proliferative capacity of aneuploid cells, in present case, these disturbances were well tolerated by proliferating cells. Furthermore, origin of trisomic genomes with both primary and tertiary chromosomes strongly indicated presence of both numerical and structural chromosomal aberrations in pollen mother cells of fasciated bud. Quite remarkably, the percentage of rolled leaf with cytological anomaly including aneuploidy increased gradually and fasciated portions invaded some new regions of stem surface following onset of flowering. This indicated some degree of added proliferation in which new regions are being affected during reproductive growth, although it is generally known that unlike animal cells plant cells cannot metastasize. Presumably, EMS-treatment induced mutations that tolerated huge cytological anomalies as well as aneuploid load and improved the fitness of multiple different aneuploidies, as advocated in budding yeast and animal tumor cells [63–65]. Induction of aneuploidy is a strong indication of cancerous growth of cells, as revealed in plant HNO cell line and also in animal cancer cell lines [5, 7]. Under influence from biotic and abiotic factors excessive multiplication of cells can lead to new plant tumor, as revealed by plant crown gall tumorigenesis [66]. Obviously, mutagenesis acted as an inducer of leaf rolling and stem as well as bud proliferations in the present* rlfL-1* mutant but whether this proliferation represents neoplastic progression in the present mutant, studies on organogenic totipotency are necessary to ascertain it.

Upon imposition of BSO treatment, significant reversals of mutant traits were noticed. Percentage of rolled-leaf phenotype and stem fasciation reduced to 1% at seedling stages and disappeared during flowering stages (Figures 5(a) and 5(b)). Bud fasciation was conspicuously absent in MuT plants (Figure 5(a)). However, premature leaf senescence coupled with necrotic spots on leaf and stem surface and significant reduction in shoot as well as root dry weight occurred in BSO-treated mutant and TM plants (Table 2; Figure 5(a)) but the damage was more pronounced in TM plants (Figure 6). Presumably, BSO-treatment inhibited tissue proliferation in the mutant plant but at the same time induced necrosis. Necrosis has been considered as initiation of death of cells and tissues and has been reported in Crown-gall tumor tissue of grapes, maize, cauliflower, and in* Arabidopsis* [67]. Typical cancer cells show susceptibility to necrosis [7]. In the present study, cell death through necrosis might be a defense mechanism of the mutant plant to suppress the proliferated tissues, as has been explained in crown-gall necrosis in different plants [67] and necrosis induced by environmental carcinogen, mutagen, virus infections, and heavy metal stress [37, 68].

### 3.2. Mitotic Fidelity in *rlfL-1* Mutant

Mitotic index (MI), duration, and transition of divisional phases are the important features of mitotic fidelity and cellular fitness [50]. Number of dividing cells and rate of cell divisions determine the rate of cell production by a meristem [21]. MI in the rolled leaf-tip of the mutant was scored fourfold higher in comparison to MC plants (Table 2). This indicated differential cellular response of proliferated cells and nonproliferated cells. This observation was further substantiated by the sharp differences in transition of divisional phases, determined by phase indices between MC and mutant leaf-tip cells. Results in Table 2 revealed that PI value was greatly reduced while MtI, AI, and TI values increased over MC values by about 3-4-fold in the rolled-leaf tips (Table 2). The results suggested that most of the cells in growing tip of rolled leaflet rapidly entered into next phase of divisions to complete the divisions, and obviously, high MI values in mutant plants might be attributed to high frequency of cells passing through these three stages. Quite alarmingly, most of the chromosomally aberrant cells in rolled leaf tips were scored in metaphase and anaphase stages, and high TI values confirmed that the dividing cells in rolled leaf tip successfully completed their divisional cycle. Duration of each phase also deviated sharply in the mutant plants from those observed in MC plants. The periodicity of divisional phases was ascertained through timewise monitoring of duration of four mitotic phases through simple fixation procedure standardized for the grass pea genotypes (Talukdar, unpublished). Total duration (prophase to telophase) was estimated to be 105 min considering peak period of particular stage in MC plants (Figure 7). Contrastingly, mean duration of total divisional phases reduced by about 2.5-fold in the mutant plants (Figure 7). Although duration of prophase and telophase changed marginally, compared to MC, peak metaphase and anaphase duration in the mutant reduced by about 3-fold and 2-fold, respectively (Figure 7), resulting in sharp decline of phase duration in rolled leaf mitotic stage. The shortening of divisional duration might be due to necessity of the mutant for a quick turnover of cell division process and carrying over high number of dividing cells (high MtI and AI values) in the next division cycle. However, this carries the high risk of newly formed aberrant cells including aneuploidy in growing leaf tips.

Dramatic turnover of mitotic events in mutant and MC plants was observed once the BSO was added in the medium. Compared to MuC, MI values reduced significantly and became close to MC value in MuT (Table 2), indicating signs of normalization of mitotic events in MuT plants. Similar situation was encountered in case of phase indices and duration of divisional stages in mutant plants. While PI value was enhanced, MtI, AI, and TI reduced considerably, reaching close to their respective MC values (Table 2). Peak metaphase and anaphase durations enhanced significantly but no significant change was observed for prophase and telophase (data not shown). In TM plants, BSO-exposure induced sharp decline in MI values which were mainly orchestrated through reduction in phase indices and duration of metaphase and anaphase. The results clearly suggested that favorable GSH-redox pool is extremely important in maintaining proper frequency, rate, and proceedings of mitotic events in plant cell and agreed well with earlier studies on* Arabidopsis rml 1, rice mil1,* and BSO-treated genotypes exhibiting huge short-fall in GSH pool [6].

### 3.3. Involvement of Cys and GSH Pool and Regulations of Gene Expressions in Controlling *rlfL-1* Phenotype

In order to ascertain the remarkable fitness of* rlfL-1* mutant despite several cytological abnormalities, roles of thiol cascade mediated by Cys and GSH were investigated. Measurable GSH levels were significantly higher in rolled leaves and fasciated stems of the mutant plants than that in MC plants. However, Cys level in mutant tissues was marginally higher than the MC level (Table 2). The GSSG pool was close to MC plants, leading to very high GSH-redox in the mutant tissues (Table 2). GSH is important in maintaining intracellular redox balance and increased GSH level was found to be associated with a proliferative response and is essential for survival of proliferative tissue through rapid cell cycle progression in both plant and animal cells undergoing tumorigenesis [5–7, 69]. In the present investigation, high mitotic activity powered by elevated frequency of dividing cells and rapid turnover during metaphase and anaphase in growing tip of rolled leaf might be the consequences of high GSH-redox, maintaining quite favorable reducing environment for cell divisions. A net increase in the total GSH pool of the dividing cells may also be required to ensure that sufficient GSH is available for distribution between the newly formed cells following mitosis, as explained in proliferating* Arabidopsis* cells [69]. This might be instrumental in maintaining and originating new fasciated portions in stems and buds of the present* rlfL-1* mutant. However, occurrence of high karyomorphological anomalies in MuC plants despite elevated GSH pool is interesting. GSH is recruited in the nucleus, and in proper redox, it is known to protect nuclear apparatus [69]. Certainly, quick turnover of cell division process and inherent instability of tumor cells led to consistent fault in chromosomal pairing and association which, accompanied by spindle disturbances as manifested by multipolarity, diagonal anaphase, laggard, and so forth in MuC plants, was inherited in the subsequent divisional stages without getting any chance to correct it properly. The importance of GSH in maintaining leaf-rolling and stem as well as bud proliferations in the present* rlfL-1* mutant was also evidenced once BSO was added in the medium. BSO is a specific inhibitor of *γ*-ECS, the first committed enzyme of GSH-biosynthesis. Measurable GSH level reduced while GSSG pool enhanced significantly in rolled leaves and fasciated stems exposed to BSO, resulting in sharp decline in GSH-redox in proliferated tissues (Table 2). Low GSH-redox severely perturbs ROS-homeostasis, tilting the delicate balance in favor of oxidative cellular environment, and triggers series of oxidative damage in plant cell [2, 3]. GSH is usually recruited by cell during early stage of cell proliferations [69], and any disturbances in its redox state towards oxidative environment may sensitize proliferative tissue towards oxidative stress. Although GSH deficiency leads to severe disturbances in plant phenotypic manifestations and ontogeny [5–8, 13], reversals of rolled leaf and fasciated stem in the present case presumably were the consequences of reduced GSH-redox status. Surprisingly enough that despite huge GSH pool in proliferating tissues of the present mutant, BSO-treatment reduced its level in a comparable amount in both proliferating and nonproliferating tissues. In order to ascertain it, a time-course preliminary analysis with BSO was conducted. The results revealed that GSH level in fasciated tissues and rolled leaf was marginally changed at initial stage of treatment but started to decline from 30 h onwards and severe depletion was measured at 120 h (Talukdar, Unpublished). Occurrence of severe necrosis coupled with premature senescence in leaves of the present mutant and in TM plants suggested that depleted endogenous GSH-pool in the proliferating tissues was unable to maintain the cell growth due to substantial loss in pace of mitotic activity. Yet, occurrence of small percentage of leaf rolling and fasciation in BSO-treated mutant at initial treatment period is important. Although there is still no evidence that GSH is synthesized in nucleus of the plant cell, substantial amount of GSH can be recruited by plant nucleus at the expense of the cytosolic GSH pool [69]. As GSH pool within nucleus is highly resistant to BSO treatment, it seems likely that high GSH level was maintained by proliferating tissues for some time which ultimately declined due to inhibition of GSH biosynthesis by BSO and continuous consumption of GSH to meet cellular demands. Remarkably enough, Cys pool was significantly higher in TM plants than MC but markedly reduced to MC level in BSO-treated MuT plants (Table 2).

Enzyme activity and gene expression analysis pointed out upregulations of mRNA transcripts controlling OAS-TL and *γ*-ECS activities in* rlfL-1* mutant (Figures 8, and 9(a)). No significant change was observed in relative expressions of two* LsSAT* isoforms (Figures 8, and 9(a)). The enhanced expression of* OAS-TL* was mainly due to increased abundance of both putative* OAS-TLA* and* OAS-TLC* transcripts (Figures 8, and 9(a)). This was concomitant with significant rise in OAS-TL activity in the mutant plants (Table 3), indicating transcriptional regulations of* OAS-TL* genes in the present grass pea mutants. Similarly, significant upregulations of  **γ*-ECS* transcripts in the mutant steered activity of *γ*-ECS enzymes by about 3.5-fold increase over MC level (Table 3). The *γ*-ECS is a rate-limiting enzyme and uses Cys as the vital building block of *γ*-glutamylcysteine, the precursor of GSH in the chloroplast [1–3]. In nonproliferating cells, high GSH level often regulated *γ*-ECS activity through feedback inhibition [2]. However, in the present mutant, stimulated Cys and GSH biosynthesis led to increased GSH accumulation presumably to keep the cells proliferating. Moreover, increased GSH synthesis in proliferating cells would serve to restore the redox potential of the cytosol and thus whole cell redox homeostasis [5, 20]. Similar role of GSH in progression of cancer was noticed in animal cells [20], although direct effect of Cys metabolisms in maintaining GSH level was not explored. The present study indicated that upstream thiol metabolisms (Cys biosynthesis) may play vital roles in keeping downstream thiol-status favorable to maintain proliferative growth in plant cell. Therefore, without ruling out other possibilities, vigorous consumption of Cys required for GSH biosynthesis might be one of the causes for marginal increase in Cys pool in MuC plants, despite high OAS-TL activity. This concept was further strengthened in BSO-treated mutant and mother plants. Compared to MuC,* OAS-TL* expressions and enzyme activity were only marginally changed but transcript abundance and activity of *γ*-ECS were not observed in MuT plants (Figures 8, and 9(a)). In TM plants, BSO treatment has no effect on* OAS-TL* gene expressions and activity but like MuT plants *γ*-ECS transcript was not detectable at all. The results reaffirmed specific inhibition of *γ*-ECS by BSO without any apparent effect on Cys-synthesizing machinery. The nonsignificant change in activity and gene expressions of both isoforms of* LsSAT* in MC, MuC, MuT, and TM plants suggested constitutive expressions of the genes during Cys biosynthesis, and thus upregulations of Cys biosynthesis in the present grass pea mutant were mainly conferred by enhanced transcripts of* OAS-TL* isoforms. The responsiveness of OAS-TL to changing cellular and physiological environment has been elucidated in* Arabidopsis*, cereals, and legumes, experiencing diverse cellular and metabolic alterations during stress [1, 4, 15]. Interestingly, Cys pool was significantly higher in TM plants than MC, MuC, and MuT despite nonsignificant change in SAT and OAS-TL activity and transcript abundance. Contrastingly, OAS-TL activity was much higher in MuT plants; yet Cys pool markedly reduced. The results strongly indicated that Cys is consumed or metabolized by way(s) other than GSH in the present* rlfL-1* mutant exposed to BSO. Certainly, this has not been operative in TM plants, resulting in Cys overaccumulation.

### 3.4. Analysis of GSH-Dependent Antioxidant Defense Response and Gene Expressions in *rlfL-1* Mutant

The rise of GSH redox pool in MuC and its substantial fall in the mutant plants upon BSO treatment has cascading effect on antioxidant gene expressions and defense response. Activities of APX, GR, GSTs, and GPX increased in both leaves and stems of MuC plants by about 2.5-, 4.2-, 5.5-, and 1.9-fold, respectively, over those in the MC plants (Table 3). By contrast, SOD activity was marginally changed in the mutant. The activities of most of the enzymes except* LsGST2* isoform were regulated at transcriptional level. Relative gene expressions of* LsAPX1*,* LsAPX2*,* LsAPX3*,* LsGr1*,* LsGr2*,* LsGST1*, and one* LsGPX* isoform were significantly upregulated in the stems and leaves of the mutant plants (Figure 8). Compared to MC, no significant change in expressions, however, was observed in* Cu/ZnSOD I* and* II* and one* FeSOD* isoform in the mutant (Figures 8, and 9(b)). APX and GR are the two important constituents of AsA-GSH cycle. With several isoforms, APX is the most prolific H_2_O_2_-scavenging machinery within cell [2, 3, 38]. On the other hand, GR has immense significance in maintaining GSH redox by regenerating GSH from its oxidized form GSSG [2, 3].* Arabidopsis* and* Lathyrus sativus* L. mutants deficient in GR activities reportedly failed to maintain proper GSH-redox value despite normal *γ*-ECS activities [2, 10]. Upregulations of gene expressions and significantly increased activities of APX and GR enzymes might be instrumental in maintaining H_2_O_2_ and GSH pool close to MC level in the mutant. The favorable GSH pool, in turn, galvanized activities of GSTs and GPX, the two prominent enzymes in intracellular detoxification system outside AsA-GSH cycle [12, 13, 41]. GST exclusively requires GSH to perform its diverse functions within cell [12, 13]. Significant overexpressions of* LsGST1* isoform and enzyme activity in rolled leaf and fasciated stem tissues suggested stimulations of GSH-mediated antioxidant defense in the proliferating tissues to contain ROS. Although GPX can use thioredoxins besides GSH as one of its electron donors [41], upregulation of its isoforms boosted antioxidant defense of mutant plants against lipid peroxides in presence of high GSH pool. Increased GPX activity using GSH as substrate was observed in an AsA-deficient mutant of grass pea [70]. In* Ctenanthe setosa* (Rose.) Eichler (Marantaceae), leaf rolling phenotype was maintained by increased activities of AsA-GSH cycle enzymes and capability of the plants to maintain high GSH-redox during cell differentiation [25]. Obviously, GSH-mediated upregulations of ROS-scavenging machinery keep ROS level under tight control in the present mutant plants, managing lipid peroxidation and membrane damage well within the limit (Table 3). The MDA content and EL% in both stem and leaf tissues of* rlfL-1* mutant hovered around the level measured in MC plants (Table 3). High ROS level accompanied by elevated level of MDA and EL% is the strong indication of oxidative damage in plant cells [2, 4, 8, 10, 11, 15, 45, 46, 69, 70]. Present results clearly pointed out absence of any such stress in the* rlfL-1* mutant.

Blockage of the GSH-mediated detoxification system enhanced the chemosensitivity of several animal tumor cell lines [5]. This enhancement was often engineered through production of excess ROS, targeting proliferated cells [5, 69]. Generation of oxidative intermediates has been proposed to be a critical event in the process of necrosis and cell death induced by various agents [5]. Consequently, depletion of GSH has been found to either precede the onset of apoptosis or render the cells more sensitive to cell death [5]. In the present study, cellular environment was dramatically changed once BSO was added in the medium. Activity and transcript abundance of SOD isoforms were enhanced by about 2–4-fold over MuC, but those of APX, GST, and GPX enzymes were reduced significantly in MuT plants (Table 3; Figures 8, and 9(b)). While APX activity reduced by about 3.8-fold, GSTs and GPX activity was lowered by nearly 4-fold and 1.5-fold, respectively, in the MuT plants (Table 3). Increased SOD activity was mainly due to enhanced transcriptional expressions of both of its* Cu/ZnSOD* and* FeSOD *isoforms. Contrastingly, downregulations to the tune of 3-4-fold in MuT plants triggered fall of APX, GST, and GPX activities to a considerable extent. The differential behavior of* LsGST2* transcript expression in relation to enzyme activity suggested possible posttranscriptional regulations of the isoform. More or less similar situation was observed in case of TM plants (Table 3; Figure 8). Increased* SOD* transcripts indicated generation of excess superoxide radicals in both stems and leaves of MuT and TM plants and response of SOD isoforms to dismutate it. Increased SOD expressions coupled with decreased activity of APX not only engineered over accumulation of H_2_O_2_ but also impeded ability of cells to scavenge it. As *γ*-ECS activity was blocked by BSO; the GSH synthesis was severely affected. This along with growing consumption of GSH to quench accumulated ROS consequently led to serious decline in GSH redox state through increased oxidation of GSH to GSSG. No significant change in GR activity and expression of its two isoforms, however, was observed in MuT and TM plants compared to their respective controls (Table 3; Figure 8). This was due to the fact that both GR isoforms expressed constitutively in presence or absence of BSO treatment. Furthermore, kinetic studies pointed out that at high GSSG concentrations, the NaDP^+^, one of the products of GR action, could act as competitive inhibitors of GR [4, 39]. This might be another reason for nonsignificant change of GR activity between BSO-treated genotypes and their untreated controls in the present case. High GSSG levels led to reduced GSH-redox in MuT and TM plants, hovering even below 0.5, despite the favorable GR activity. Certainly, maintenance of GSH-redox by GR was insufficient to meet the growing demand for GSH. Low GSH pool seriously jeopardized effectiveness of GST and GPX activities and thereby caused serious impediment in scavenging of toxic cell metabolites and peroxides. The resultant excess accumulation of ROS consequently led to high rate of membrane damage through elevated level of lipid peroxidation in MuT and TM plants (Table 3), marking the onset of oxidative stress. ROS-triggered oxidative damage was manifested by marked decline in plant dry weight and severe necrosis in leaves and stems of both MuT and TM plants. Although traditionally necrotic cell death is considered unprogrammed and uncontrolled, recent study in animal and plant cells revealed that its occurrence might be tightly regulated [71], and ROS may play an important role in determining necrosis [71]. In several crop plants and* Arabidopsis*, oxidative burst led by elevated H_2_O_2_ level caused cell death through necrosis during* Agrobacterium*-mediated transformations [67]. In the present study, to get more insights regarding involvement of ROS in cell proliferation and necrosis, a pilot experiment was carried out using thiourea (TU, a ROS-scavenger) in the medium with or without BSO. Surprisingly enough, magnitude of leaf rolling and stem fasciation reduced to 60% of MuC plants in TU-treated mutant, whereas no necrosis was observed on stem and leaf surface of BSO + TU-treated mutant (Talukdar, unpublished). Primary analysis pointed out drastic reduction of H_2_O_2_ level even below MC plants in rolled leaves (mean 1.12 ± 0.5) and fasciated stem (mean 0.98 ± 0.05) of the TU-treated mutant. In BSO + TU-treated mutant, H_2_O_2_ level also declined from MuC level but was very close (mean 3.32 ± 0.8) to that measured in MC. It seems likely that along with high GSH level, cells must have certain H_2_O_2_ level to maintain proliferations. Its reduction to MC level in BSO + TU-treated mutant was certainly enough to abolish necrosis and cell death. The results indicated that delicate balances of ROS are the determining factor for cell proliferations and necrosis, of course, in the presence of favorable GSH-redox to go either way. The dual roles of H_2_O_2_ as an inducer of ROS-mediated oxidative damage as well as cell death and also a signaling molecule to upregulate antioxidant defense to withstand oxidative stress have been studied during plant-pathogen interactions, legume-rhizobium symbiosis, tolerance to abiotic stresses, and in diverse metabolic and cellular events of plant growth and development [9–11, 20, 37, 44]. Present results confirmed coordinated expressions of antioxidant defense in generating mutant phenotypes and its reversal through necrosis which is sensitive to the redox state of the cell, determined by glutathione pool and the generation of the oxidant H_2_O_2_ within cell [3, 4, 9, 71].

### 3.5. BSO Treatment Reveals Metabolic Diversion through Cys and Its Cascading Effect on Oxidative Metabolisms of *rlfL-1* Mutant

In order to ascertain the possible reasons behind high Cys level in TM plants and its reduction to MC level in MuT plants, we studied desulfuration of Cys predominantly catalyzed by LCD and DCD. Activities of both the enzymes were substantially lower in MuC plants than MC (Table 3). However, compared to MuC, activities of LCD and DCD were enhanced by about 4.0-fold and 3.5-fold, respectively, in leaves and stems of MuT plants (Table 3). This enhancement was mainly due to transcriptional overexpressions of* LsLCD* and* LsDCD* genes in MuT leaves and stems (Figures 8, and 9(a)). By contrast, no significant change in relation to MC was observed in transcripts abundance and concomitant enzyme activity in TM plants (Table 3; Figures 8, and 9(a)). As H_2_S is the major product of LCD and DCD activities, endogenous H_2_S levels were measured in MuT and TM plants. A 3–3.5-fold increase in H_2_S content was observed in MuT tissues while no such effect was noticed in TM plants (Table 3). The results clearly pointed out consumption of Cys through upregulations of its degradation pathway in MuT plants in view of the inhibition of GSH biosynthesis, resulting in reduction of Cys content to MC level in MuT plants exposed to BSO. Although Cys is the vital building blocks of proteins and numerous cellular functions, growing evidence indicates that Cys-homeostasis is fundamental for plant metabolisms and unregulated accumulation of free Cys, but not GSH, over a certain threshold can act as powerful prooxidant within plant cell [16, 17]. Diversion of Cys metabolic route through its sulfuration in the present MuT plants was, therefore, unique and was not observed in TM plants, leading to overaccumulation of Cys but very low H_2_S content in latter case. H_2_S can act as a gaseous signaling molecule in promotion of plant growth and stress tolerance [18, 19, 43], but over certain level it can induce oxidative stress through generation of increased ROS by modulating plant photosynthesis [42]. One of such enzymes is glycolate oxidase (GO) which catalyzes oxidation of glycolate to glyoxylate during photorespiration in higher plants with the production of H_2_O_2_ [4, 42]. Compared to MuC, GO activity increased by 3-fold (Table 3) while* GO* transcripts enhanced by about 2.5–3-fold in MuT leaves (Figures 8, and 9(c)). The results suggested that transcriptional upregulations of* GO* genes conferred increased enzyme activities in BSO-treated mutant plants. No significant change in gene expressions and enzyme activity was observed in TM plants in relation to MC (Table 3; Figures 8, and 9(c)). It is thus noteworthy that a blockage in GSH-synthesizing machinery not only hampered GSH-redox pool but also triggered significant changes in cellular ROS metabolisms through diversions of Cys metabolisms and concomitant induction of* GO* gene presumably by H_2_S in MuT plants. Obviously, high GO activity accompanied with elevated SOD and low APX might be instrumental in accumulation of excess H_2_O_2_ and consequent oxidative damage of membrane in MuT plants. H_2_S-induced ROS-mediated cell death has been reported, although in delayed responses in wheat aleurone cells [72].

### 3.6. ROS Imaging by CLSM Study

The differential mode of ROS accumulation in leaves and stems of MC, MuC, MuT, and TM was strongly evidenced by ROS imaging study by CLSM. In MC and MuC, slight red fluorescence due to superoxide radicals localized only in epidermal region was detected (Figures 10(a) and 10(b)). The magnitude of red fluorescence, however, was markedly increased in leaves and stems of MuT and TM plants (Figures 10(c)–10(e)). In leaves of MuT plants, the red fluorescence was detected in high amount in and around vascular regions, sclerenchyma, mesophyll, and epidermis (Figures 10(c) and 10(e)). When the leaf and stem sections were preincubated with 1 mM TMP (a superoxide scavenger), a significant reduction of the fluorescence was observed (Figures 10(f) and 10(g)), thus exhibiting the specificity of DHE for detection and imaging of superoxide radicals in grass pea tissues. For H_2_O_2_ imaging, cross section of MC and MuC leaves and stems incubated with DCF-DA exhibited a bright green fluorescence which was restricted to only epidermis and xylem regions of vascular tissue and additionally in sclerenchyma region of MuC leaves (Figures 10(h) and 10(i)). In leaves and stems of MuT and TM plants, the green fluorescence was enhanced markedly in vascular bundles, sclerenchyma, mesophyll regions (leaf), and in epidermis (Figures 10(j)–10(l)). A preincubation with 1 mM ascorbate considerably tamed the florescence (Figures 10(m) and 10(n)). The analysis of superoxides and H_2_O_2_ by CLSM showed an enhanced generation of superoxide radicals and H_2_O_2_/other peroxides and their abundant localizations in leaf and stem tissues of MuT and TM, exposed to BSO. Overproduction of superoxides and H_2_O_2_ was distinctly visible by CLSM study in crop plants [2, 3, 37]. The absence of both red and green fluorescences in mesophyll tissues of present MC and MuC and their abundant occurrence even in overlapping conditions with tissue autofluorescence (blue) in some cases in leaves of MuT and TM plants suggested involvement of chloroplasts in ROS production in the present materials. Both red and green fluorescences were considerably tamed in plants treated with thiourea (Figures 10(o)–10(r)), a ROS-scavenger. The results confirmed that BSO treatment strongly induced ROS generation in both* rlfL-1* mutant and its mother variety and both superoxide generations and H_2_O_2_ productions are regulated by fine tuning of antioxidant defense in the present* rlfL-1* mutant.

## 4. Conclusions 

The* rlfL-1* mutant exhibited characteristic leaf-rolling and stem as well as bud fasciation in grass pea. Both the phenomena were associated with severe disturbances in chromosomal behavior including origin of aneuploidy and were powered by vigorous mitotic cell divisions, indicating cell proliferations and tolerance to unbalanced genomes. Coordinated overexpressions of vital Cys and GSH-synthesizing genes and upregulations of GSH-dependent antioxidant defense under favorable GSH-redox in MuC leaves and stems contained ROS within MC level, as imaged by CLSM study. Several unique events were detected once BSO was added to the medium. Reversal of mutant phenotypes occurred in association with significant downregulations of GSH-synthesis and concomitant reduction of GSH-redox as well as GSH-dependent antioxidant defense, resulting in overaccumulation of ROS and onset of severe necrosis in MuT. These events were accompanied by upregulations of genes involved in Cys-desulfuration, release of H_2_S, and overexpressions of GO in photorespiratory pathway in MuT but not in TM. Presumably, onset of necrosis coupled with premature leaf senescence during BSO-mediated reversal of rolled leaf and stem fasciation in the present mutant involves (1) downregulations of GSH-mediated antioxidant capacity, (2) upregulations of Cys-degrading pathways and induction of more H_2_O_2_ production through H_2_S, and (3) ROS-mediated onset of cell death via necrosis. Results indicated that high GSH-redox pool is vital in maintaining leaf-rolling and fasciation and ROS-mediated cell death through diversion of excess Cys-pool to H_2_S production during reversal of the mutant traits. Occurrence of multiple nucleoli per cell, aneuploidy, and susceptibility to necrosis strongly suggested cancerous nature of the present mutant traits. Present results revealed intricate relationships between cell biological parameters and events controlled by thiol-redox particularly Cys and GSH in proliferating plant cells and can be utilized in future research regarding ROS-signaling in plant cell proliferation through H_2_O_2_-H_2_S relationships and concomitant cellular and metabolic responses.

## Figures and Tables

**Figure 1:** (a) Normal linear-lanceolate leaflets in a compound leaf of mother variety BioL-212, (b) inwardly leaf rolling in* rlfL-1* mutant, (c) commencement of leaf rolling in* rlfL-1* mutant, and (d) initiation of normal leaflet in mother variety BioL-212 at early seedling stage.

**Figure 2:** (a) Mother plant BioL-212 with flower bud (→) and nonfasciated stem, (b) mutant* rlfL-1* with rolled leaflet, fasciated stem (thick arrow), and fasciated drooping buds (thin arrow) in field condition.

**Figure 3:** (a) Normal 2*n* = 2*x* = 14 chromosomes in leaf-tip cells of mother variety BioL-212, (b) unoriented abnormal metaphase, (c) aneuploid cells with 2*n* = 2*x* + 1 = 15 chromosomes, (d) C-mitosis, (e) C-mitotic chromosomes undergoing breakage, (f) mitotic cytomixis, (g) unoriented aneuploid metaphase, (h) sticky metaphase, (i) anaphase bridge broken, (j) anaphase delayed, (k) anaphase bridge with or without laggard (→), and (l) diagonal orientation at late anaphase in dividing leaf-tip cells of* rlfL-1* mutant. Bar represents 1 SD = 10 *μ*m.

**Figure 4:** (a) Normal seven bivalents in meiotic metaphase I in pollen mother cells of mother variety BioL-212, (b) six bivalents and two univalents (→) at metaphase I, (c) unoriented 14 chromosomes at anaphase I, (d) long retention of double nucleoli (→) at anaphase I, (e) double nucleoli at diakinesis (→), (f) “Y”-shaped trivalents (→) in trisomic diakinesis, (g) one pentavalent (thick arrow) and one univalent (thin arrow) in trisomic diakinesis, (h) two trivalents (→) and three bivalents in diploid diakinesis, (i) one quadrivalent (thin arrow) and one trivalent (thick arrow), two univalents and three bivalents in a trisomic metaphase I, (j) seven bivalents and one univalent in trisomic metaphase I, (k) one trivalent (→), one univalent, and five bivalents in diploid metaphase I, (l) one rod-shaped trivalent (thin arrow), two univalents (thick arrow), and five bivalents in a trisomic metaphase I, (m) unequal 8-7 chromosome separation at anaphase I, (n) anaphase bridge with lagging chromosome (→), (o) broken anaphase bridge (→), (p) micronuclei (→) at telophase II in pollen mother cells of fasciated buds of* rlfL-1* mutant. Bar represents 1 SD = 10 *μ*m.

**Figure 5:** (a) and (b) Reversal of leaf rolling and stem as well as bud fasciation (→) accompanied with occurrence of necrosis and yellowing of leaves (→) in BSO-treated* rlfL-1* mutant of grass pea.

**Figure 6:** A BSO-treated mother (TM) variety BioL-212 and its mutant (MuT)* rlfL-1* exhibiting leaf and stem necrosis and premature leaf senescence symptoms.

**Figure 7:** Duration of mitotic phases in* rlfL-1* mutant (M) and its mother variety BioL-212 in grass pea. Bar followed by error bar represents means ± SE of at least four replicates.

**Figure 8:** mRNA gene expression analysis of* Lathyrus sativus* (Ls) serine acetyl transferases (SATs) 1;1 and 1;2, O-acetylserine thiol lyase (OAS-TL) A and C, *γ*-glutamylcysteine synthetase (*γ*-ECS), Cu/Zn superoxide dismutase (SOD) I and II, FeSOD, ascorbate peroxidase (APX) 1, 2, and 3, glutathione reductase (Gr) 1 and 2, glutathione* S*-transferase (GST) 1 and 2, glutathione peroxidase (GPX), L-cysteine desulfhydrase (LCD), D-cysteine desulfhydrase (DCD), and glycolate oxidase (GO) isoforms in lanes 1,3,5,7-leaves of mother control (MC), mutant control (MuC), BSO-treated mutant (MuT), and BSO-treated mother (TM), respectively, and in lanes 2,4,6,8-stems of MC, MuC, MuT, and TM plants, respectively, by qRT-PCR, followed by 2% agarose gel electrophoresis with* EF1-*α** used for cDNA normalization and a 100 bp DNA marker (M) (arrow 300 bp).

**Figure 9:** Relative expressions of genes governing mRNA transcripts of* Lathyrus sativus* L. (a) thiol-metabolizing enzymes and isoforms of SAT, OAS-TL, *γ*-ECS, LCD, and DCD; (b) antioxidant defense genes controlling SOD, APX, GR, GST, and GPX isoforms; (c) GO in leaves (L) and stems (St) of MC (mother control), MuC (mutant control), BSO-treated* rlfL-1* mutant (MuT), and BSO-treated mother (TM). The mRNA levels were normalized with respect to housekeeping gene* EF-1*α** and are expressed relative to those of control (MC) value, which were arbitrarily given a value of 1. Data are means ± SE of five biological replicates and two technical replicates. Asterisks denote significant changes (upregulation and downregulation) of genes with respect to control values.

**Figure 10:** Representative imaging of superoxide radicals and H_2_O_2_ productions in* Lathyrus sativus *L. leaves by CLSM. Images are developed from several optical sections collected by confocal microscopy showing the autofluorescence (blue; excitation at 633 nm, emission at 680 nm) and fluorescence due to DHE and DCF-DA. Superoxide-dependent DHE fluorescence (red) in leaf cross sections from (a) mother control, (b) mutant control, (c) BSO-treated mutant, (d) BSO-treated mother with blue autofluorescence, and (e) stem cross section from BSO-treated mutant; ((f), (g)) for the negative control, leaves (f) and stems (g) of mutant were incubated with 1 mmTMP, a superoxide scavenger; ((h)–(n)) H_2_O_2_-dependent DCF-DA fluorescence (green) in leaf cross sections of (h) mother control, (i) mutant control, (j) BSO-treated mother, (k) BSO-treated mutant, and (l) stem cross section of BSO-treated mutant; ((m), (n)) as a negative control, leaves were incubated with 1 mm ascorbate (ASC), which acts as a H_2_O_2_ scavenger in BSO-treated (m) mother and (n) treated mutant, (o) stem cross section of stem and (p) leaves of thiourea + BSO-treated mutant with DHE fluorescence (red), (q) thiourea + BSO-treated leaves, and (r) stems of mutant with H_2_O_2_-dependent DCF-DA fluorescence (green). The results are representative of at least three independent experiments. Ep: epidermis; Hp: hypodermis; Ms: mesophyll cells; Scl: sclerenchyma; Xy: xylem vessels. Bars = 50 *μ*m.

**Table 1:** Oligonucleotide primers used in qRT-PCR analysis of the expression of selected target genes in grass pea (*Lathyrus sativus* L.) genotypes. F: forward, R: reverse primers.

Target genes	Primers (5′→3′)	Amplicon size (bp)
*LsSAT1;1 *	F-GGCCATACTTATTCTATCTCTGAGTG-	317
	R-AACAGTATATGTACTCTCAGCAGTAAC-	
*LsSAT1;2 *	F-GGACCATATTTCCATCTCTGAGTG-	287
	R-CTACTAGCAATAATCAACCTTTTCATC-	
*OAS-TLA *	F-CTCACAAGATTCAAGGGATAGGA-	397
	R-GTCATGGCTTCCGCTTCTTTC-	
*OAS-TLC *	F-GATCCTACCGCAGTGTCTGAACGAAA-	406
	R-GACGTCTCACAATTCTGGCTTCAT-	
*Ls*γ*-ECS *	F-CAGCTTAGTGGTGCACCATCTTGA-	171
	R-TGCTCAAACCCAAAAGTTAAC-	
*LsGST 1 *	F-GATATTCTGGGCTTGGATTTTGT-	161
	R-GTTCTCTCCCAACTCTCCTTGCT-	
*LsGST 2 *	F-CTTGGTCCTCCTCCGCTAACT-	156
	R-GAAAGTCCTCCTCCGCTAACT-	
*LsGPX *	F-ACTATGGCTGCCCCCACAT-	118
	R-TCTGGCATCTTTGACGGTGA-	
*LsLCD *	F-TCACTACGCAAACGGAGCACA-	139
	R-TCATTATTCACCGCCATCACC-	
*LsDCD *	F-GGATAGGAGGCATCCAAAGC-	156
	R-TAAGATTAAACGTTCAACCAAGA-	
*Cu/Zn SOD I *	F-CCGTTCCATATCCATGCCGGT-	305
	R-AGCTACTCTGCCACCAGCAT-	
*Cu/Zn SOD II *	F-AAGCATTTCAACTGGACCAG-	224
	R-TTCCACCTTTCCCAAGAGAT-	
*Fe SOD *	F-CCGACCACAGAGCTTATGTA-	213
	R-GAGTGGATGATGATGGTT-	
*LsAPX 1 *	F-AACTTGGCCCTGGCGTTGTTGCT-	239
	R-CAGAACCGTCCTTGTAAGTGC-	
*LsAPX 2 *	F-ATGGAGAGTGAAGGCAAAGCAT-	220
	R-CGCAGTCAAGCTCGCATACGATA-	
*LsAPX 3 *	F-GGACTCCAGCCGATCAAAGA-	208
	R-CGAACATTGGTCAGGTCCAG-	
*LsGr1 *	F-TGATATTGCTAGTCTGTATGCGT-	212
	R-CAGGAACTCCAAGGCACAATGT-	
*LsGr2 *	F-AGTCTGCTCTTCACGTAGACCG-	192
	R-GTTGGCTGTGGGTGATGTCCGAA-	
*LsGO *	F-CTTATGTCTTTCGCTGTTGCCAGATA-	139
	R-AGATATGCTGTTACATTTCCGTTAA-	
*EF1-*α** (Housekeeping)	F-ATTTCGACTCTGGGAAGTCAA-	198
	R-ATCTTTACTATTTCAGCCTTA-	

**Table 2:** Phenotypic characteristics, cytological peculiarities, and biochemical features in *rlfL-1* mutant and its mother variety Biol-212 under untreated and BSO-treated conditions. MC-untreated (no BSO) mother control, MuC-untreated (no BSO), MuT-BSO-treated mutant, and TM-BSO treated mother plant.

Traits	MC	MuC	MuT	TM
Shoot dry weight (g plant^−1^)	0.16 ± 0.02^b^	0.29 ± 0.03^a^	0.10 ± 0.02^c^	0.07 ± 0.008^c^
Root dry weight (g plant^−1^)	0.19 ± 0.03^b^	0.34 ± 0.03^a^	0.12 ± 0.04^b^	0.06 ± 0.007^c^
Pod length (cm)	3.38 ± 0.35^b^	5.87 ± 0.49^a^	3.41 ± 0.39^b^	1.21 ± 0.12^c^
100 seed weight (g)	5.85 ± 0.43^b^	11.85 ± 0.53^a^	5.90 ± 0.44^b^	2.37 ± 0.37^c^
Seeds pod^−1^	3.56 ± 0.13^a^	3.07 ± 0.11^a^	1.15 ± 0.09^b^	1.21 ± 0.13^b^
Pollen sterility (%)	1.33 ± 0.32^c^	43.11 ± 0.53^b^	45.51 ± 0.61^b^	63.77 ± 0.71^a^
MI%	15.51 ± 0.56^b^	61.05 ± 0.77^a^	15.63 ± 0.61^b^	7.56 ± 0.19^c^
PI%	70.33 ± 0.67^b^	2.53 ± 0.11^c^	66.67 ± 0.57^b^	80.93 ± 0.67^a^
MtI%	17.97 ± 0.32^b^	51.17 ± 0.45^a^	18.63 ± 0.32^b^	7.37 ± 0.32^c^
AI%	8.69 ± 0.11^b^	31.30 ± 0.39^a^	10.69 ± 0.11^b^	7.09 ± 0.11^c^
TI%	3.01 ± 0.10^b^	13.00 ± 0.17^a^	4.01 ± 0.10^b^	4.61 ± 0.10^b^
Cysteine content (nmoL g^−1^ FW) leaf	7.43 ± 0.54^b^	9.19 ± 0.54^b^	7.51 ± 0.59^b^	33.89 ± 0.67^a^
Cysteine content (nmoL g^−1^ FW) stems	6.89 ± 0.33^b^	7.03 ± 0.34^b^	6.77 ± 0.59^b^	29.76 ± 0.63^a^
GSH (nmoL g^−1^ FW) leaf	73.5 ± 4.8^b^	257.8 ± 7.7^a^	1.93 ± 0.09^c^	1.87 ± 0.11^c^
GSSG (nmoL g^−1^ FW) leaf	11.7 ± 1.1^c^	12.9 ± 2.1^c^	222.8 ± 6.3^b^	228.3 ± 4.1^a^
GSH redox-leaf (GSH/(GSH + GSSG))	0.863 ± 0.07^b^	0.954 ± 0.08^a^	0.008 ± 0.00^c^	0.008 ± 0.00^c^
GSH (nmoL g^−1^ FW) stems	70.5 ± 4.3^b^	247.9 ± 7.9^a^	1.95 ± 0.09^c^	1.90 ± 0.11^c^
GSSG (nmoL g^−1^ FW) stems	12.7 ± 1.1^b^	12.8 ± 2.1^b^	225.9 ± 6.6^a^	230.3 ± 4.7^a^
GSH redox-stems (GSH/(GSH + GSSG))	0.847 ± 0.09^b^	0.951 ± 0.09^a^	0.008 ± 0.00^c^	0.008 ± 0.00^c^

Data are means ± SE of at least four replicates. Means followed by same alphabets are not significantly (*P* > 0.05) different at ANOVA followed by Duncan's multiple range test. MI: mitotic index, PI: prophase index, MtI: metaphase index, AI: anaphase index, TI: telophase index, GSH: reduced glutathione, and GSSG: glutathione disulfide.

**Table 3:** Activities of *γ*-glutamylcysteine synthetase (*γ*-ECS, nmol min^−1^ g^−1^ FW), serine acetyl transferase (SAT, U mg^−1 ^protein), O-acetylserine thiol lyase (OAS-TL, nmol cysteine min^−1^ mg^−1 ^protein), superoxide dismutase (SOD, U min^−1^ mg^−1^ protein), ascorbate peroxidase (APX, µmol ascorbate oxidized min^−1^ mg^−1^ protein), glutathione reductase (GR, nmol NADPH oxidized min^−1^ mg^−1^ protein), glutathione-S transferases (GSTs, U mg^−1^ protein), and glutathione peroxidase (GPX, nmol NADPH min^−1^ mg^−1^ (protein)), L-cysteine desulfhydrase (LCD, nmol H_2_S min^−1^ mg^−1 ^protein), D-cysteine desulfhydrase (DCD, nmol H_2_S min^−1^ mg^−1 ^protein), hydrogen sulfide level (H_2_S, µmol g^−1^ FW) and glycolate oxidase (GO, µmol glyoxylate min^−1^ mg^−1^ protein) H_2_O_2_ (µmol g^−1^ FW), malondialdehyde (MDA, nmol g^−1^ FW) in *rlfL-1* mutant and its mother variety Biol-212 under untreated and BSO-treated conditions.

Traits	MC	MuC	MuT	TM
*γ*-ECS	6.8 ± 1.1^b^	23.8 ± 4.2^a^	ND	ND
SAT	0.65 ± 0.08^a^	0.69 ± 0.05^a^	0.64 ± 0.03^a^	0.64 ± 0.07^a^
OAS-TL	23.6 ± 1.97^b^	70.2 ± 3.33^a^	69.7 ± 3.12^a^	22.5 ± 1.90^b^
SOD-leaf	180.3 ± 9.1^b^	178.9 ± 6.3^b^	359.7 ± 10.5^a^	356.6 ± 10.6^a^
SOD-stems	165.3 ± 7.3^b^	170.7 ± 5.9^b^	343.4 ± 9.5^a^	350.8 ± 11.0^a^
APX-leaf	131.3 ± 8.8^b^	328.3 ± 11.2^a^	34.56 ± 2.4^a^	35.66 ± 1.9^a^
APX-stems	111.5 ± 6.7^b^	282.3 ± 11.2^a^	29.67 ± 2.8^c^	30.59 ± 2.5^c^
GR-leaf	31.2 ± 2.2^b^	131.04 ± 12.5^a^	129.8 ± 12.3^a^	30.9 ± 2.1^b^
GR-stems	33.2 ± 2.2^b^	134.07 ± 10.8^a^	130.9 ± 12.9^a^	33.9 ± 2.8^b^
GSTs-leaf	0.22 ± 0.08^b^	1.21 ± 2.8^a^	0.30 ± 0.08^b^	0.05 ± 0.008^c^
GSTs-stem	0.25 ± 0.10^b^	1.25 ± 2.9^a^	0.33 ± 0.07^b^	0.06 ± 0.008^c^
GPX-leaf	7.1 ± 0.98^b^	13.49 ± 3.3^a^	8.99 ± 0.89^b^	4.72 ± 0.77^c^
GPX-stems	7.8 ± 0.99^b^	12.87 ± 3.2^a^	9.01 ± 0.90^b^	4.69 ± 0.69^c^
LCD-leaf	20.38 ± 0.64	11.67 ± 0.45	46.67 ± 0.78	19.38 ± 0.63
LCD-stems	17.54 ± 0.45^b^	10.58 ± 0.39^c^	37.03 ± 0.41^a^	18.54 ± 0.41^b^
DCD-leaf	16.15 ± 0.63^b^	9.87 ± 0.37^c^	40.23 ± 0.69^a^	16.03 ± 0.59^b^
DCD-stems	13.18 ± 0.55	7.99 ± 0.29	28.01 ± 0.72	13.20 ± 0.51
H_2_S level-leaf	0.047 ± 0.003^b^	0.029 ± 0.002^c^	0.087 ± 0.006^a^	0.050 ± 0.003^b^
H_2_S level-stems	0.033 ± 0.002^b^	0.025 ± 0.001^c^	0.088 ± 0.007^a^	0.034 ± 0.002^b^
GO activity-leaf	0.85 ± 0.03^b^	0.76 ± 0.03^b^	2.28 ± 0.09^a^	0.83 ± 0.02^b^
H_2_O_2_-leaf	3.32 ± 0.81^c^	3.19 ± 0.62^c^	21.67 ± 0.98^a^	14.56 ± 0.34^b^
H_2_O_2_-stem	3.21 ± 0.67^c^	3.05 ± 0.62^c^	17.13 ± 0.54^a^	10.44 ± 0.29^b^
MDA-leaf	4.23 ± 0.71^c^	4.13 ± 0.65^c^	28.78 ± 0.87^a^	16.23 ± 0.33^b^
MDA-stems	3.99 ± 0.53^c^	3.20 ± 0.44^c^	22.56 ± 0.49^a^	14.31 ± 0.29^b^
EL%-leaf	4.04 ± 0.38^c^	4.16 ± 0.38^c^	27.34 ± 0.55^a^	12.87 ± 0.22^b^
EL%-stems	3.87 ± 0.29^c^	4.10 ± 0.35^c^	25.58 ± 0.50^a^	12.32 ± 0.19^b^

Data are means ± SE of at least four replicates. Means followed by same alphabets are not significantly (*P* > 0.05) different at ANOVA followed by Duncan's multiple range test. MC-untreated (no BSO) mother control, MuC-untreated (no BSO), MuT-BSO-treated mutant, and TM-BSO treated mother plant.
